# Seroconfirmed Typhoid Fever and Knowledge, Attitude, and Practices among Febrile Patients Attending at Injibara General Hospital, Northwest Ethiopia

**DOI:** 10.1155/2021/8887266

**Published:** 2021-04-13

**Authors:** Wondemagegn Mulu, Chalachew Genet Akal, Kidist Ababu, Solomon Getachew, Fenkil Tesfaye, Asamrew Wube, Desalegn Chekol

**Affiliations:** Department of Medical Laboratory Science, College of Medicine and Health Science, Bahir Dar University, Ethiopia

## Abstract

**Introduction:**

Typhoid fever (TF) is a febrile global health problem caused by *Salmonella enterica* serovar Typhi (*S.* Typhi) with relatively high prevalence in low- and middle-income countries including Ethiopia. Identifying local prevalence and gaps in knowledge, attitude, and practice (KAP) towards TF is recommended by the World Health Organization to implement preventive measures. Therefore, this study determined the prevalence of *S*. Typhi and KAP of febrile patients towards TF in Injibara General Hospital, Northwest Ethiopia.

**Methods:**

Hospital-based cross-sectional study was conducted from January to March 2020. A total of 237 patients were included conveniently. Data on KAP and demographic variables were collected using a structured questionnaire by face-to-face interview. After the interview, 5 ml venous blood was collected and processed using the Widal test following the manufacturer's instruction. Mean scores and percentages were used to determine the level of KAP. Multivariable analysis was done to correlate KAPs with TF. *P* value < 0.05 was considered statistically significant.

**Results:**

The overall prevalence of *S*. Typhi was 25.7%. The highest seroprevalence was observed among the age group of 30-34 years (33.3%) and patients with no education. The majority of participants know the major ways of TF transmission (59.1-90.7%) and prevention (81.4%) methods. However, the misconception on the route of TF transmission was observed in 13.5-36.7% of participants. About 65.4% and 67.5% of study participants were considered knowledgeable and had good preventive practice towards TF, respectively. Being a student (AOR = 0.227, CI = 0.053 − 0.965) and considering mosquito bite as transmission routes (AOR = 2.618, CI = 1.097 − 6.248) were significantly associated with TF.

**Conclusion:**

High *S*. Typhi prevalence was observed in the study area. Moreover, the misconception on the transmission of typhoid fever and educational level was a risk factor for TF. Thus, health facilities should incorporate topics on typhoid fever as part of their health education system within health facilities and in the community.

## 1. Introduction

Typhoid fever (TF) is a febrile life-threatening disease caused by the bacterium *Salmonella enterica* serovar Typhi (*S.* Typhi). *S*. Typhi, where humans are the only host and reservoir, is mainly transmitted through the fecal-oral route [1]. Typhoid fever is a global health problem [1] which causes around 11-21 million cases and 128, 000-161 000 deaths annually where the majority of cases and deaths occurring in Asia and sub-Saharan Africa largely driven by lack of access to clean water and poor sanitation [1–7]. Moreover, recent studies done on the burden of TF in low- and middle-income countries revealed an increasing trend of TF in Africa [2, 3, 8, 9].

Though different laboratory test methods and clinical specimens are used, the prevalence of *S*. Typhi is variable among different countries in Africa [9] and among different geographical locations in Ethiopia [10]. Previous studies done showed a heterogeneous prevalence of *S*. Typhi in African countries ranging from 5%–69.6% [11–15]. Similarly, TF, one of the major public health problems, showed 5%-56.2% *S*. Typhi prevalence at different times and geographical areas of Ethiopia [16–21].

The burden of *S*. Typhi is affected by different geographical areas, times, persons, and places [8]. Besides lack of access to safe water, poor sanitation, poor handwashing practices (after using toilet, before eating food, and before preparing food), eating raw foods (milk, vegetables, and meat), improper disposal of human and other wastes, close contact with TF cases or carriers, and low level of education increased the risk of acquiring *S*. Typhi [1, 21–24].

As indicated by World Health Organization (WHO) [1] and other studies [8, 16, 22], TF can be prevented by maintaining food safety, safe water supply, proper sanitation, vaccination, and health education to create public awareness and induce behavioral change after identifying knowledge, attitude, and practice (KAP) gaps and by adapting it to local conditions in the study area.

Knowledge is necessary to acquire optimum health. Attitude development is not essentially a function of the amount of information one receives but a function of how that information was acquired. Furthermore, advancing the knowledge of communities towards TF is a powerful means to foster favorable attitude and exercising preventive practices among the population. Therefore, a clear understanding about the knowledge, attitude, and practices (KAPs) among any community is required to interrupt and prevent the transmission of TF. Determining the prevalence of *S*. Typhi, KAPs of the community towards TF, and identifying associated factors on TF will have paramount importance to implement proper TF prevention and control strategies. Thus, the present study was intended to determine the seroprevalence of *S*. Typhi and KAP of febrile patients towards TF in Injibara general hospital, Northwest Ethiopia.

## 2. Materials and Methods

### 2.1. Study Design, Setting, and Period

A hospital-based cross-sectional study was conducted in Injibara General Hospital from January to March 2020. Injibara General Hospital has 145 beds serving around 1.2 million people. The hospital is found in Injibara town, the largest town of Awi zone found in Amhara regional state, Ethiopia. The town is located 120 kilometers (km) and 431 km away from the region capital Bahir Dar and country capital Addis Ababa, respectively.

### 2.2. Source and Study Population

The source population was all febrile patients attending Injibara General Hospital in the study period. Febrile patients clinically diagnosed for TF in the study period were considered as the study population.

### 2.3. Inclusion and Exclusion Criteria

#### 2.3.1. Inclusion Criteria

All patients having signs and symptoms of TF including fever, headache, malaise, abdominal discomfort, and giving written informed consent were included.

#### 2.3.2. Exclusion Criteria

Patients clinically diagnosed as TF suspects but unconscious during the study period were excluded.

### 2.4. Sample Size and Sampling Technique

A total of 237 study participants were included using a single population proportion formula taking 19% prevalence of *S*. Typhi from a study done in Amhara regional state, Ethiopia [20], 5% margin of error, and 95% level of confidence. A convenient sampling method was used to enroll study participants. Any patients who fulfilled the inclusion criteria were included consequently until the required number was achieved.

### 2.5. Data Collection, Clinical Sample Processing, and Serological Testing

All febrile patients visiting the Injibara General Hospital outpatient department (OPD) were examined clinically by physicians, and those presumptive for TF were requested for a Widal test. After getting written informed consent, data on KAP and demographic variables were collected by face-to-face interview using a structured questionnaire which was pretested in Tibebe-Ghion Specialized Hospital. After the interview, a 5 ml blood specimen was collected from each study participant in the Injibara General Hospital laboratory department using a test tube without anticoagulant. The collected blood was processed to get serum, and the Widal slide agglutination test was done to detect *S*. Typhi using known *S*. Typhi flagella (H) and somatic (O) antigen (Linear Chemicals. S. L. U., Barcelona, Spain) following the manufacturer's instructions.

### 2.6. Scoring of KAP Questions

Twelve, 2, and 9 questions were used to assess the knowledge, attitude, and preventive practices of study participants towards TF, respectively. Study participants who gave the right response on KAP questions were given a score of 1, and those who did not were given 0 score. The score of each study participant obtained out of 12, 2, and 9 for knowledge, attitude, and practice questions, respectively, was summed up separately. A mean value for each knowledge, attitude, and practice questions was calculated. Study participants scoring the mean or above the mean value were considered knowledgeable or had favorable attitudes or good practice.

### 2.7. Quality Control

Before data collection, the questionnaire was pretested and every questionnaire was cheeked for its completeness after collection. Standard bacteriological procedure and manufacturer's instruction were followed during specimen processing and performing Widal test. A positive and negative control test was performed along with the test specimen.

### 2.8. Data Analysis

Collected data were entered and analyzed using Statistical Package for Social Science 23 (IBM Corp Released 2011.IBM SPSS statistics. Armonk, NY: IBM Corp). Descriptive statistics such as mean score and percentage were computed to determine the magnitude of KAPs and background variables. Chi-square test and logistic regression analysis were done to determine factors associated with seroprevalence of *S*. Typhi and *P* value < 0.05 was considered as statistically significant.

### 2.9. Ethical Considerations

Ethical clearance was obtained from the Institutional Review Board (IRB) of Bahir Dar University, College of Medicine and Health Sciences. Moreover, before data collection, permission letter and written informed consent were obtained from Injibara General Hospital and each study participant, respectively.

## 3. Results

### 3.1. Demographic Characteristics of Study Participants

Among 237 febrile patients included, 128 (54%) were females. The mean age of the study participants was 33 years. Moreover, the majority of study participants was married (53.2%) and completed at least secondary education (56.5%) (Table 1).

### 3.2. Prevalence of *S*. Typhi

The overall seroprevalence of *Salmonella* Typhi (reactive at least for H or O antigen) was 25.7%. Among 61 seropositive study participants, 41 (67.2%) were positive for O-antigen, and the rest 12 (19.7%) and 8 (13.1%) were positive for H-antigen and for both H and O antigen, respectively. The highest *S*. Typhi seroprevalence was observed among the participant age group of 30-34 years, patients with no education, and rural residents with 33.3%, 37.3%, and 32.1%, respectively (Table 1).

### 3.3. Knowledge of Study Participants towards Typhoid Fever

The study also assessed the knowledge, attitude, and practice of study participants on typhoid fever causative agent, transmission, and prevention methods. Among 12 questions asked, the overall mean score for correctly answered knowledge questions was 9.8 ± 1.6. One hundred fifty-five (65.4%) scored mean and above the mean and considered to be knowledgeable while 82 (34.6%) scored below the mean and considered as not knowledgeable towards TF. With no statistically significant difference, the prevalence of *S*. Typhi among knowledgeable and not knowledgeable study participants towards TF were 25.2% and 26.8%, respectively, (COR = 1.091, CI = 0.593 − 2.004).

About 44.7% of study participants did not know that typhoid fever is caused by microorganisms. More than 90% and 86% of study participants know that typhoid fever can be transmitted by contaminated food and contaminated water, respectively. On the other hand, 36.7% and 13.5% of participants have a misconception that typhoid fever can be transmitted by respiratory droplets and mosquito bite, respectively. Majority of study participants know the common typhoid prevention methods including proper food cooking (93.2%) and washing fruits and vegetables (88.6%) (Table 2).

### 3.4. Attitude and Preventive Practice of Study Participants towards Typhoid Fever

Two attitude and 9 preventive practice questions were used for assessing study participants' attitude and preventive practices towards TF, respectively. The overall mean score of study participants' attitude towards TF was 1.2 ± 0.5. Though not significant, the prevalence of TF was higher in study participants having poor attitudes (27.7%) than those having favorable attitudes (18.9%) towards TF (COR = 1.649, CI = 0.771 − 3.526). The overall mean score of the participant preventive practice level was 6.9 ± 1.2. Study participants who had good and poor preventive practice towards TF were 160 (67.5%) and 77 (32.5%), respectively. With no statistically significant difference, the prevalence of *S*. Typhi among study participants having good and poor preventive practice towards TF were 25.6% and 26%, respectively (COR = 1.018, CI = 0.547 − 1.895).

Almost all (98.7%) of the study participants perceived that typhoid fever is a preventable disease. Though the overall practice on possible ways of TF prevention is low (68, 28.7%), the majority of the study participants implement the main preventive practices of washing hands before having meals (96.6%) and after using the toilet (94.9%). Moreover, the seroprevalence of *S*. Typhi was significantly higher among study participants who did not implement all six prevention practices listed (29.6%) than those who did (16.2%) (*P* = 0.003). Though 73.4% of study participants believe that they are not exposed to different infection sources for TF, majority of study participants consume raw vegetables (85.2%), raw meat (66.7%), and lack garbage can in their houses for waste collection (58.6%). The study also indicated that 95.4% and 76.4% of study participants used homemade food and pipe water, respectively (Table 3).

### 3.5. Multivariable Analysis on Risk Factors of *S*. Typhi Seroprevalence

On multivariable analysis, typhoid fever was significantly associated with educational level and considering mosquito bite as a transmission route. Study participants who considered mosquito bite as a means of TF transmission had 2.6 times more chance to have TF compared with those who did not consider mosquito bite as a transmission means. Even though it was not significant, higher seroprevalence was found in study participants who used river water (27.1%) (*P* = 0.811) and consumed restaurant foods (36.4%) than those who used pipe water (25.4%) and consumed homemade foods (25.2%), respectively (Table 4).

## 4. Discussion

The prevalence of *S*. Typhi in the present study was 25.7%. Based on the 2016 demographic and health survey of Ethiopia [25], there is a low rate of availability of water and soap for handwashing among households. The availability was lowest in Amhara regional state (5%) where the present study was conducted. This poor availability of water and soap can contribute to the high prevalence of TF in the present study. The prevalence of the present study was comparable with the study done in India [26].

On the other hand, the prevalence of TF in the present study is much higher than studies done in other parts of Ethiopia such as West Gojjam zone [18], Gondar [20], Shashemene [17], and Amibara [19] reporting 5.8%, 19.1%, 5%, and 13.2%, respectively. Moreover, it was also higher than studies done outside of Ethiopia including Kilosa District, Tanzania [11], Papua New Guinea [14], Egypt [15], and Indonesia [24] reporting 10.3%, 8%, 5%, and 9%, respectively. These variations in the burden of TF might be because of an increase in TF through time which is supported by different studies [9] and low specificity of Widal test [1] coupled with the possibility of multiple febrile infection occurrences as reported in different studies done in Ethiopia [18, 20].

On the other hand, the prevalence of TF in the present study was lower than a study done in West Wollega [27] and Ambo [21], Ethiopia, which reported 53.6% and 56.2% *S*. Typhi infection, respectively. These variations might be due to study participant differences in terms of KAP towards typhoid fever. Moreover, known HIV and inpatients were included in other studies, which might increase the seroprevalence. Similarly, the seroprevalence in the present study was lower than a study done in Nigeria among university students [13] reporting 69.6%. This variation might be due to the difference among study participants where students from Nigeria were living in a single campus, which might allow the occurrence of high TF prevalence in a specific study period because of a common infection source.

In the present study, 155 (65.4%) and 160 (67.5%) study participants were knowledgeable and have good preventive practice towards TF, respectively. Having secondary and above educational level was significantly associated with being knowledgeable (*P* = 0.002) and good preventive practice (*P* = 0.017) towards TF. On the other hand, only 53 (22.4%) of the study participants have a favorable attitude towards TF. Moreover, attending high-level education was not significantly associated with having a favorable attitude (*P* = 0.118).

About 98.7% of the study participants know that TF is a preventable disease. This was higher than a study done in West Wollega, Ethiopia [27], reporting 76.1%. This difference might be because of the study period and educational level difference of study participants where in the present study 22.3% have an educational level above secondary school unlike a study in West Wollega, Ethiopia [27]. Moreover, 94.9% and 41.4% of the study participants practiced handwashing after toilet and have garbage can for waste collection in their house, respectively. This was higher than a study done in West Wollega, Ethiopia [27], reporting 71.4% for handwashing practice after toilet and 12.1% for garbage can. This variation might be because of a higher percentage of employed study participants in the present study giving them an economical advantage.

Majority of study participants believed that eating contaminated food (90.7%) and drinking contaminated water (86.1%) are means of TF transmission in the present study. Similarly, on TF prevention practices, handwashing before meals (96.2%) and after using the toilet (96.2%) was reported. This finding was comparable with a study done in Burundi [28].

In the present study, 91.1% of study participants have a toilet, which is comparable with a study in Tanzania (95%) [22]. On the other hand, 78.5%, 45.1%, and 81.4% of study participants had aware of TF signs, possible transmission methods, and prevention methods, respectively. This finding was higher than a study done in Tanzania [22]. These might be because of study period differences, which might increase the present study participants' access to health information.

The source of drinking water and food for 76.4% and 95.4% of study participant was pipe water and homemade food, respectively, in the present study. This was comparable with the 2016 Ethiopian DHS report [25]. Though not significant, the higher seroprevalence of *S*. Typhi was indicated in the study participants using river water (27.1%, *P* = 0.811) and restaurant foods (36.4%) (*P* = 0.409) than using pipe water (25.4%) and homemade foods (25.2%), respectively. A comparably high seroprevalence but the significantly associated finding was reported in Shashemene, Ethiopia [17], with source of water and food and in Ambo, Ethiopia [21], with source of water.

There was no significant associate of raw meat consumption with seroprevalence of *S*. Typhi. But these were in contrary with a study done in Ambo, Ethiopia [21], where raw meat consumption was significantly associated with seroprevalence. This variation might be because of geographical differences contributing for different hygienic and food consumption practices. Moreover, in the present study, there was no significant association of seroprevalence with not having a toilet in their house (*P* = 0.756). But this was in contrary to a study done in Jakarta, Indonesia, where not having a toilet was significantly associated with the prevalence of *S*. Typhi [24]. This variation might be linked with environmental differences among the study area.

The study had few limitations. Because of test limitations associated with Widal agglutination test including cross-reaction of antibodies produced against *S*. Typhi O and H antigen with other Enterobacteriaceae coupled with false-positive results in patients with malaria and other infections [1], the study might not indicate the actual prevalence of *S*. Typhi in the study area. Furthermore, since the study was hospital-based, it might not reflect the actual TF prevalence and KAP of the community on TF.

## 5. Conclusion

Despite the majority of the study participants being knowledgeable and having good preventive practice towards TF, a high prevalence of *S*. Typhi was observed in the study area. Educational level and misconception on the transmission of TF were factors associated with the existence of TF. Thus, health facilities should incorporate topics on TF as part of their health education system within the health facility and in the community in a more enhanced way. Moreover, further culture-based studies are recommended to get a better image on *S*. Typhi prevalence.

## Figures and Tables

**Table 1:** Prevalence of *S*. Typhi TF and demographic characteristics of febrile patients presumptive to have typhoid fever at Injibara General Hospital, Northwest Ethiopia, 2020.

Variables	*S*. Typhi serological test result for febrile patients (*n* = 237)		
	Nonreactive: *n* (%)	Reactive: *n* (%)	Total
Age (years)			
≤19	9 (75)	3 (25)	12
20-24	37 (72.5)	14 (27.5)	51
25-29	35 (74.5)	12 (25.5)	47
30-34	22 (66.7)	11 (33.3)	33
35-39	22 (81.5)	5 (18.5)	27
40-44	19 (82.6)	4 (17.4)	23
45-49	16 (76.2)	5 (23.8)	21
>49	16 (69.6)	7 (30.4)	23
Sex			
Male	82 (75.2)	27 (24.8)	109
Female	94 (73.4)	34 (26.6)	128
Marital status			
Never married	32 (78)	9 (22)	41
Married	91 (72.2)	35 (27.8)	126
Living together	37 (78.7)	10 (21.3)	47
Divorced/separated	10 (71.4)	4 (28.6)	14
Widowed	6 (66.7)	3 (33.3)	9
Educational status			
No education	37 (62.7)	22 (37.3)	59
Primary education	35 (79.5)	9 (20.5)	44
Secondary education	43 (76.8)	13 (23.2)	56
More than secondary	61 (78.2)	17 (21.8)	78
Residence			
Rural	76 (67.9)	36 (32.1)	112
Urban	100 (80)	25 (20)	125
Occupation			
Student	43 (79.6)	11 (20.4)	54
Farmer	57 (64.8)	31 (35.2)	88
Merchant	31 (91.2)	3 (8.8)	34
Government employee	45 (73.8)	16 (26.2)	61
Total	176 (74.3)	61 (25.7)	237

Note: TF: typhoid fever; NR: nonreactive to *S*. Typhi serological test result; R: reactive to *S*. Typhi serological test result.

**Table 2:** Knowledge towards typhoid fever causative agent, transmission, and prevention methods among febrile patients at Injibara town, Northwest Ethiopia, 2020.

Variables	Response (*n* = 237)	
	Yes: *n* (%)	No: *n* (%)
TF causative agent and sign		
(1) TF is caused by microorganism	131 (55.3)	106 (44.7)
(2) Fever is one sign of TF	186 (78.5)	51 (21.5)
(3) TF can kill infected individuals	149 (62.9)	88 (37.1)
(4) TF is preventable disease	234 (98.7)	3 (1.3)
Know 4 listed points on TF disease, causative agent and sign	48 (20.3)	189 (79.7)
TF transmission methods & infection source		
(5) TF can be transmitted from infected person to other person	140 (59.1)	97 (40.9)
(6) TF is transmitted by eating contaminated food	215 (90.7)	22 (9.3)
(7) TF is transmitted by drinking contaminated water	204 (86.1)	33 (13.9)
(8) TF carriers can act as source of TF infection	160 (67.5)	77 (32.5)
Know four listed transmission method and infection source	107 (45.1)	130 (54.9)
TF prevention methods		
(9) Handwashing before meal can prevent TF	228 (96.2)	9 (3.8)
(10) Handwashing after using toilet can prevent TF	228 (96.2)	9 (3.8)
(11) TF can be prevented by proper food cooking	221 (93.2)	16 (6.8)
(12) TF can be prevented by washing fruits and vegetables	210 (88.6)	27 (11.4)
Know four listed TF prevention methods	193 (81.4)	44 (18.6)
Misconceptions on TF transmission		
(1) TF is transmitted by respiratory droplets	87 (36.7)	150 (63.3)
(2) TF is transmitted by mosquito bite	32 (13.5)	205 (86.5)
Knowledge questions (*n* = 12 questions)		
Mean knowledge score = 9.8 (Min = 1, Max = 12)		
Overall knowledge status (*n* = 237)		
Knowledgeable = 155 (65.4%)		
Knot knowledgeable = 82 (34.6%)		

Note: TF: typhoid fever; Min: minimum; Max: maximum.

**Table 3:** Attitude towards typhoid fever and preventive practice on TF among febrile patients at Injibara town, Northwest Ethiopia, 2020.

Variables	Response (*n* = 237)	
	Yes: *n* (%)	No: *n* (%)
Attitude related questions		
(1) Do you believe yourself as exposed to TF infection source	63 (26.6)	174 (73.4)
(2) Do you believe TF is a preventable disease	205 (86.5)	33 (13.9)
TF prevention practices questions		
(1) Do you wash your hand after using toilet	225 (94.9)	12 (5.1)
(2) Do you wash your hand before meal	229 (96.6)	8 (3.4)
(3) Do you wash hands before preparing food	231 (97.5)	6 (2.5)
(4) Do you consume raw fruits and vegetables	202 (85.2)	35 (14.8)
(5) Do you consume raw milk	108 (45.6)	129 (54.4)
(6) Do you consume raw meat	158 (66.7)	79 (33.3)
Practice all above six TF prevention practices	68 (28.7)	169 (71.3)
(7) Do you have garbage can for waste collection at home	98 (41.4)	139 (58.6)
(8) Do you have toilet	216 (91.1)	21 (8.9)
(9) Do you have pipe water	181 (76.4)	56 (23.6)
Attitude questions (*n* = 2 questions)		
Mean attitude score = 1.1 (Min = 0, Max = 2)		
Overall attitude status (*n* = 237)		
Favorable attitude = 53 (22.4%)		
Unfavorable attitude = 184 (77.6%)		
Preventive practice question (*n* = 9 questions)		
Mean attitude score = 6.9 (Min = 2, Max = 9)		
Overall preventive practice status (*n* = 237)		
Good preventive practice = 160 (67.5%)		
Poor preventive practice = 77 (32.5%)		

Note: TF: typhoid fever; Min: minimum: Max: maximum.

**Table 4:** Multivariable analysis on the associated factors of *S*. Typhi among febrile patients at Injibara General Hospital, Northwest Ethiopia, 2020.

Variable	Seroprevalence of *S*. Typhi		AOR (95% CI)	*P* value
	Nonreactive: *n* (%)	Reactive: *n* (%)		
Educational status (*n* = 237)				
No education (*n* = 59)	37 (62.7)	22 (37.3)	1.428 (00.523-3.897)	0.487
Primary education (*n* = 44)	35 (79.5)	9 (20.5)		0.636
Secondary education (*n* = 56)	43 (76.8)	13 (23.2)	0.711 (0.173-2.924)	0.937
More than secondary (*n* = 78)	61 (78.2)	17 (21.8)	1.060 (0.247-4.559)	
			1	
Occupation (*n* = 237)				
Student (*n* = 54)	43 (79.6)	11 (20.4)	0.227 (0.053-0.965)	0.045
Farmer (*n* = 88)	57 (64.8)	31 (35.2)	1.506 (0.376-6.026)	0.563
Merchant (*n* = 34)	31 (91.2)	3 (8.8)	0.518 (0.177-1.519)	0.231
Government employee (*n* = 61)	45 (73.8)	16 (26.2)	1	
TF can be caused by mosquito bite (*n* = 237)				
Yes (*n* = 32)	19 (59.4)	13 (40.6)	2.618 (1.097-6.248)	0.030
No (*n* = 205)	157 (76.6)	48 (23.4)	1	
Hand washing after using toilet (*n* = 237)				
Yes (*n* = 225)	170 (75.6)	55 (24.4)	1	
No (*n* = 12)	6 (50)	6 (50)	2.099 (0.521-8.468)	0.297
Washing hand before food preparation (*n* = 237)				
Yes (*n* = 231)	174 (75.3)	57 (24.7)	1	
No (*n* = 6)	2 (33.3)	4 (66.7)	6.846 (0.862-54.382)	0.069
Waste collection system available (*n* = 237)				
Yes (*n* = 98)	77 (78.6)	21 (21.4)	1	
No (*n* = 139)	99 (71.2)	40 (28.8)	1.303 (0.632-2.685)	0.474
TF can kill if untreated (*n* = 237)				
Yes (*n* = 149)	112 (75.2)	37 (24.8)	1	
No (*n* = 88)	64 (72.7)	24 (27.3)	5.227 (0.560-48.791)	0.147

Note: TF: typhoid fever.

## Data Availability

Since all data was provided in the article, no more data will be uploaded.

## Abbreviations

KAP: Knowledge, attitude, and practice
OPD: Outpatient department
TF: Typhoid fever
WHO: World Health Organization.
